The article "Study on the Influencing Mechanism of Human Chorionic Gonadotropin (hCG) on Oocyte Maturation in Patients with Polycystic Ovary Syndrome" was retracted in 2023. Reasons: suspected computer-generated content; unreliable results or conclusions; concerns about the data; concerns about the results or conclusions.

# Study on the Influencing Mechanism of Human Chorionic Gonadotropin (hCG) on Oocyte Maturation in Patients with Polycystic Ovary Syndrome

**DOI:** 10.1155/2022/7933166

**Published:** 2022-07-14

**Authors:** Jingjing Jiang, Shanshan Gao, Ting Han

**Affiliations:** Center for Reproductive Medicine, Shandong University, No. 157 Jingliu Road, Jinan, 250021 Shandong, China

## Abstract

The study was aimed at investigating the influence of human chorionic gonadotropin (hCG) hormone on oocyte maturation in the patients with polycystic ovary syndrome (PCOS). A total of 54 patients with PCOS who received *in vitro* maturation (IVM) treatment in the Cheeloo College of Medicine, Shandong University, were divided into two groups: one group who underwent hCG injections was the observation group (OG; *n* = 27) and other was the control group (CG; *n* = 27) with no hCG injection. The oocyte development and the expression of steroid hormone synthesis-related genes including gonadotropin-releasing hormone receptor (GnRHR), Conexin43, epidermal growth factor-related genes, luteinizing hormone/choriogonadotropin receptor (LHCGR), epiregulin (EREG), and vascular endothelial growth factor (VEGF) were examined. The human ovarian granulosa cell line (SVOG cells) and ovarian epithelial cell line (HOSEpiC cells) were employed to analyze the effect of hCG on the biological behaviour of cells. As a result, OG showed higher normal fertilization, cleavage, and high-qualified embryo rate than CG. Expression levels of GnRHR, Cx43, LHCGR, EREG, and VEGF were significantly elevated in granulosa cells in the OG group. Western blot revealed that phosphoinositide 3-kinase (PI3K), protein kinase B (AKT), and rapamycin (mTOR) proteins were decreased in granulosa cells under hCG intervention. A biological behaviour test indicated that the multiplication capacity of hCG-intervened SVOG and HOSEpiC was increased, while the apoptosis was decreased. In conclusion, hCG could accelerate follicular development and oocyte maturation by activating oocyte maturation genes in PCOS patients, which could significantly improve and popularize the application of IVM technology.

## 1. Introduction

Polycystic ovary syndrome (PCOS) is an endocrine disease, prone to occur in women during the reproductive age, with main symptoms of menstrual disorders and infertility [1–3]. According to statistics, PCOS-caused infertility accounts for approximately 50%-70% of ovulatory infertility [4]. *In vitro*-assisted reproductive technology is recommended to PCOS patients complicated with tubal obstruction, pelvic adhesion, and endometriosis [5]. However, many PCOS patients are susceptible to ovulation drugs and some may even develop ovarian hyperstimulation syndrome (OHSS), which threatens their safety in severe cases [6, 7]. At present, the uncontrollable ovarian response, OHSS, and the quality of oocytes in patients with PCOS after ovulation induction are still the difficulties and hotspots in the field of assisted reproductive technology [8].

*In vitro* maturation (IVM) technology is an effective treatment method that immature granulosa cell-oocyte complexes are retrieved from antral follicles [9]. IVM technology will increase the oocyte maturation rate in PCOS patients and reduce the occurrence of OHSS [10, 11], which will also help to achieve a sufficient number of high-quality oocytes. However, due to the unsatisfactory effect caused by the failure of oocyte maturation, most patients need the injection of human chorionic gonadotropin (hCG) hormone [12]. hCG is a glycoprotein secreted by trophoblast cells of the placenta, an effective diagnostic index for several diseases during pregnancy, and a hormone nourishing the specific growth and metabolism of somatic cells [13, 14]. The effects of hCG on oocytes have been clarified [15], but the underlying mechanisms remain elusive.

Accordingly, this study preliminarily explored the underlying mechanism of the effects of hCG on pregnancy outcomes in IVM patients via detecting the expression levels of granulosa cell oocyte maturation-related genes in PCOS patients, providing a theoretical basis for treatment alternatives and prognosis judgment in clinical practice.

## 2. Materials and Methods

### 2.1. Patient Information

A total of 54 patients with PCOS who received IVM in the Center for Reproductive Medicine Affiliated to Shandong University from January 2019 to June 2019 were included in this study and divided into the following two groups: one is the observation group (OG; *n* = 27) where hCG injections were given to patients to promote ovulation, and the other is the control group (CG; *n* = 27) where no hCG injection was given. The study was approved by the Ethics Committee of Reproductive Medicine of Shandong University, and all patients signed the informed consent form.

### 2.2. Inclusion and Exclusion Criteria

Inclusion criteria were as follows: patients aged more than 18 years old, who complied with the diagnostic guidelines for PCOS and underwent IVM treatment [16], and with no drug or surgical treatment in the last three months. Exclusion criteria were as follows: patients with endometriosis, thyroid disease, hyperprolactinemia, thrombosis adrenal, mental illness, chromosomal abnormalities, and allergic reaction to hCG injection or PCOS patients during pregnancy or lactation.

### 2.3. Intervention Measures and Sample Collection

On the menstrual cycle days 9 to12, transvaginal ultrasound scans were repeated to monitor follicle development and ensure that there were no follicles larger than 8 mm. The patients in the OG group were given an injection of hCG (Livzon Pharmaceutical Group Inc., State Drug Approval Document Number H44020673, specification: 2000 U), with a dosage of 6000-10, 000 Uimst. 36 h after injection, the follicles smaller than 10 mm in diameter were utilized for oocyte pick-up and follicular fluid and granulosa cell collection through transvaginal ultrasound guidance with the usage of an aspiration needle. In the CG group without HCG injection, oocytes were retrieved directly. In addition, 4 mL of venous blood was sampled from the patients, centrifuged to collect the serum, and kept at -80°C.

### 2.4. *In Vitro* Maturation

After oocyte pick-up, the oocytes in OG and CG groups were cultured in IVM medium containing TCM-199 medium (Sigma, USA), 0.75 U/mL FSH, 0.1 U/mL streptomycin/penicillin, and 10% FBS at 37°C in an incubator containing 5% CO_2_ for 28-32 h. After the first polar body appears, the mature oocytes in metaphase II (MII) were fertilized by intracytoplasmic sperm injection (ICSI). Fertilization was evaluated by the appearance of two pronuclei. The *in vitro* culture results of the two groups were compared, including the number of MII oocytes, metaphase I (MI) oocytes, and geminal vesicle (GV) oocytes. In embryo scoring, the scoring standard of cleavage embryos on the 3rd day was established by combining the Peter cleavage-stage embryo scoring system with the actual situation of our center. Grade I and II embryos were defined as high-quality embryos. The MII oocyte ratio, ICSI fertilization rate, cleavage rate, and rate of excellent embryos were calculated as per the below-mentioned formulae:

(1) $$\begin{array}{c} \text{MII oocyte ratio}=\frac{\text{number of MII oocytes}}{\text{Total oocytes }\left(\text{MII oocytes}+\text{MI oocytes}+\text{GV oocytes}\right)}\times 100,\\ \text{ICSI fertilisation rate}=\frac{\text{fertilized oocyte number}}{\text{ MII oocyte number}}\times 100,\\ \text{Cleavage rate}=\frac{\text{fertilized cleavage embryo number}}{\text{number of fertilized oocytes}}\times 100,\\ \text{Rate of excellent embryos}=\frac{\text{number of high}‐\text{quality embryos }}{\text{numbers of fertilized oocytes}}\times 100. \end{array}$$

### 2.5. Hormone and Growth Factor Determination

The follicular fluids of OG and CG were centrifuged. The supernatant was collected to determine follicular fluid E_2_, insulin growth factor-I (IGF-I), and hCG levels using the automatic chemiluminescence method.

### 2.6. Gene Expression Analysis

Total RNA was extracted from granulosa cells using the Trizol reagent (Invitrogen, USA) according to the standard protocol, and the concentration and quality of RNA samples were evaluated using a NanoDrop 2000 spectrophotometer (Thermo, USA). Reverse transcription was performed using the MasterMix kit (Takara, Japan). Universal SYBR Green Master Mix (Applied Biosystems, USA) was used to carry out quantitative polymerase chain reaction (qPCR) on StepOnePlus real-time PCR system (Applied Biosystems). Gene expression was normalized to GAPDH. The relative expression levels of steroid hormone biosynthesis-related genes gonadotropin-releasing hormone receptor (GnRHR) and Conexin43 (Cx43) and epidermoid growth factor-related genes luteinizing hormone/chorionic gonadotropin receptor (LHCGR), epiregulin (EREG), and vascular endothelial growth factor (VEGF) were calculated using the 2^−ΔΔCT^ method [17]. The primer sequences are listed in Table 1.

### 2.7. Cell Culture

The human ovarian granulosa cell line SVOG and ovarian epithelial cell line HOSEpiC were purchased from the American Type Culture Collection (ATCC). SVOG was cultured in Dulbecco's modified Eagle medium : Nutrient Mixture F-12 (DMEM/F-12) (Gibco BRL) containing 10% fetal bovine serum (FBS) and 1% penicillin-streptomycin in a humid environment at 37°C with 5% CO_2_ in air, while HOSEpiC cells were maintained in DMEM (Gibco BRL) plus 10% FBS and 1% penicillin-streptomycin. The logarithmic growth phase cells were seeded on the 96-well plate, and the hCG group cultured with hCG and the blank group cultured with the same amount of normal saline were set up. Both groups were cultured for 24 h, and the final concentration of hCG was 100 ng/mL.

### 2.8. Cell Proliferation Test

After the relative culture, we added 3-(4,5-dimethylthiazol-2-yl)-2,5-diphenyltetrazolium bromide (MTT, 5 mg/mL, 20 *μ*L, Beyotime Biotechnology, Shanghai, China) to each well at 0, 24, 48, and 72 h, followed by another incubation for 4 h. After 2 h of incubation with 150 *μ*L DMSO, the supernatant from the wells was collected and observed at 490 nm using a microplate analyzer to visualize the cell growth curve.

### 2.9. Apoptosis Assay and Western Blot

Apoptosis level was detected by Annexin V/propidium iodide (PI) staining (eBiosciences, USA). After 72 h transfection, the cells (5 × 10^5^) were collected and washed twice with PBS. The cells were suspended in 500 *μ*L binding buffer and then added with 5 *μ*L each of Annexin V/FITC and PI for 15 min incubation at room temperature. Attune NxT flow cytometry (Thermo Fisher Scientific, China) was used for analysis.

Cells were lysed using a lysis buffer containing a mixture of protease inhibitors (Wuhan Elabscience Biotechnology Co., Ltd., China). Protein concentration was determined by dioctinic acid assay. Then, 20 *μ*g of protein extract was isolated by sodium dodecyl sulfate-polyacrylamide gel electrophoresis (SDS-PAGE) and blotted onto a polyvinylidene fluoride (PVDF) membrane. After that, the PVDF membrane was sealed with 5% milk for 1 h and incubated with primary antibodies at 4°C overnight. After washing for 3 times, the membrane was incubated with an HRP-conjugated secondary antibody. Enhanced chemiluminescent reagent (ECL) luminescence was utilized to develop the color, and the relative protein level was calculated by ImageJ software.

### 2.10. Statistical Analysis

SPSS22.0 statistical software was employed for data analysis. The continuous variables conforming to normal distribution were expressed as means ± SD. The categorical data, recorded as *n* (%), were analyzed by the chi-square test. Student's *t*-test tested the continuous variables conforming to normal distribution. Those that did not follow normal distribution were tested by the Mann-Whitney *U* test. The Pearson coefficient was used to analyze the correlation. A probability (*p*) level less than 0.05 was set as the statistical significance.

## 3. Results

### 3.1. Comparison of General Data

The comparison showed that the two groups were not significantly different in general data such as age, BMI, educational level, residence, marital status, family medical history, contraceptive pill intake history, dietary habit, exercise habit, smoking, and history of gestation, indicating that there was comparability (*p* > 0.05; Table 2).

### 3.2. Oocyte's Maturation and Fertilization Rate

The number of MII oocytes and maturation rate were increased in the OG group after IVM treatment compared with the CG group (*p* < 0.05), while the number of MI oocytes and GV oocytes was lower (*p* < 0.05). Moreover, the OG group has a higher normal fertilization rate, cleavage rate, and high-qualified embryo rate than CG following ICSI insemination (*p* < 0.05; Figure 1 and Table 3). Overall, the maturation, cleavage, and normal fertilization rates were higher in the OG group than in the CG group.

### 3.3. Hormone and Growth Factor Determination Results

Serum IGF-I and hCG and follicular fluid E_2_, IGF-I, and hCG levels were higher in OG when compared with CG (*p* < 0.05). According to Pearson correlation coefficient analysis, hCG in serum and follicular fluid was positively correlated with E_2_ and IGF-I concentrations in OG (*p* < 0.05; Figure 2).

### 3.4. Effect of hCG on the Biological Behaviour of Ovary Cells

Cell proliferation of SVOG and HOSEpiC cells is shown in Figures 3(a) and 3(b), indicating the higher multiplication capacity of OG. Apoptosis analysis showed that cell apoptosis level was induced in the CG group (*p* < 0.05; Figure 3).

### 3.5. Expression Profiles of Mature Genes in Granulosa Cells

Significantly upregulated mRNA expression levels of mature genes, including GnRHR, Cx43, LHCGR, EREG, and VEGF, were found in granulosa cells in OG compared with CG (*p* < 0.05; Figure 4).

### 3.6. Correlation of hCG with Mature Genes

Pearson correlation coefficient analysis revealed that the concentration of hCG (21.69 ± 4.55 ng/mL) in ovarian granulosa cells in OG was positively correlated with GnRHR, Cx43, LHCGR, EREG, and VEGF mRNA levels (*p* < 0.05; Figure 5).

### 3.7. Expression of PI3K/AKT/mTOR Pathway Proteins in Granulosa Cells

Detection of the proteins related to the PI3K/AKT/mTOR pathway in granulosa cells revealed that the protein levels of PI3K, AKT, and mTOR in OG were elevated compared with those in the CG group (*p* < 0.05; Figure 6).

## 4. Discussion

Follicular development involves the interaction of oocytes, granulosa cells, and theca cells [18–20]. During the development of follicles into the secondary follicles, granulosa cells secrete mucopolysaccharides to surround oocytes and form a zona pellucida, which forms a wide gap junction with the oocytes for the transfer of nutrients and small molecules, as well as to carry out transmission and transduction [21, 22]. Therefore, a full understanding of the role of hCG in follicular activation may be the key to improving IVM success in the future.

In this study, we observed the IVM of oocytes after hCG injection. The results exhibited that the hCG intervention significantly increased the number of MII oocytes, fertilization rate, and high-quality embryo rate in OG, suggesting that hCG could facilitate follicle development and oocyte maturation. In other words, hCG functioned in promoting the aromatic transformation of androgen into estrogen and stimulating the production of progesterone [23]. Due to the essential role of estrogen and progesterone in the process of follicular development and maturation [24], we preliminarily inferred that hCG induced oocyte development by stimulating the production of estrogen and progesterone. Thus, E_2_ and IGF-I levels in patients were tested and the results revealed higher E_2_ and IGF-I in the OG group than in the CG group, indicating that E_2_ and IGF-I in patients were elevated by hCG intervention. E_2_, as the principal physiological estrogen in vertebrates, was vital in the feminine reproductive system [25]. IGF-I is an active protein polypeptide secreted during the physiological process of growth hormone, which is also a hallmark of metabolism acceleration [26]. hCG has been confirmed to promote the secretion of E_2_ and IGF-I in some diseases, such as endometritis and hysteromyoma [27, 28], which was consistent with our results.

Next, the relationship between hCG, E_2_, and IGF-I was determined through the correlation analysis, and we found that both E_2_ and IGF-I increase as the concentration of hCG increases. *In vitro* experiments also demonstrated that the activation of ovarian granulosa cells and epithelial cells significantly boosted under hCG intervention, suggesting that hCG might also modulate ovarian granulosa cells for oocyte maturation. Granulosa cells are essential in follicular development and oocyte maturation. Moreover, granulosa cells affect oocyte development and maturation by secreting various cytokines and steroid hormones in an autocrine and paracrine manner [29]. These influencing factors included transforming growth factor (TGF-*β*) superfamily, epidermal growth factor, insulin-like growth factor family, fibroblast growth factor family, cytokine family, VEGF, tumour necrosis factor, and interleukin [30]. In addition to mutual regulation, these factors in the ovary were regulated by gonadotropins [31]. Furthermore, they could modulate ovarian function through the specific receptors and change follicular response to gonadotropins. Ovarian autocrine and paracrine factors are also critical in several reproductive diseases [32]. Hence, we detected follicle maturation-related genes including GnRHR, Cx43, LhCGR, EREG, and VEGF under the intervention of hCG, and the results revealed the higher parameters in OG in comparison to CG. GnRH, sex steroid hormone, inhibin, and activin are all of great significance in regulating the expression of the GaRH receptor [33]. Cx43 played an important role in oocyte meiosis and follicular selection [34]. LHCGR could stimulate the secretion of testosterone [35]. EREG and VEGF were classic epidermal and vascular growth factors [36]. The increase in the above-mentioned genes under the intervention of hCG validated the role of hCG as a potent hormone in enhancing follicular development and oocyte maturation to preliminarily affect oocytes through the above molecular mechanisms. Previous studies elucidated the role of hCG in the activation of the PI3K/AKT/mTOR pathway [31, 37], a pathway with an essential regulatory capacity for lipid metabolism [38]. During oocyte maturation, the enhanced activation of granulosa cells led to the accelerated lipid metabolism and mass production of life-active substances, such as proteins and mitochondria, which caused the growth and maturation of oocytes [39]. Therefore, we speculated that the action pathway of hCG in granulosa cells might also be related to the PI3K/Akt/mTOR pathway. Additionally, we found that PI3K, AKT, and mTOR proteins in granulosa cells in OG were notably increased through protein detection, suggesting that the PI3K/AKT/mTOR pathway was activated, which was in line with the previous studies. Since there were only 54 patients included in this study, the results might be not comprehensive enough and need further validation.

## 5. Conclusion

The present study revealed the role of hCG in oocyte maturation-related genes in the patients with PCOS. hCG hormone increased the mRNA expression levels of the genes related to oocyte maturation in PCOS patients by activating the PI3K/AKT/mTOR pathway and accelerating follicular development and oocyte maturation, which was conducive to promoting the application of hCG hormone in IVM technology.

## Figures and Tables

**Figure 1:** Oocyte maturation: (a) comparison of the number of MII eggs; (b) comparison of the number of MI eggs; (c) comparison of the number of GV eggs. ^∗^*p* < 0.05.

**Figure 2:** Nucleic acid test results. (a) Comparison of E_2_ concentration. (b) Comparison of IGF-1 concentration. (c) Comparison of hCG concentration. ^∗^*p* < 0.05. (d) The correlation between hCG and E_2_ in serum (*r* = 0.632). (e) The correlation between hCG and E_2_ in follicular fluid (*r* = 0.654). (f) The correlation between hCG and IGF-1 in serum (*r* = 0.625). (g) The correlation between hCG and IGF-1 in follicular fluid (*r* = 510).

**Figure 3:** The effect of hCG on the biological behavior of ovarian cells: (a) SVOG growth curve; (b) HOSEpiC growth curve; (c) cell apoptosis rate. ^∗^*p* < 0.05.

**Figure 4:** Mature gene expression in granulosa cells: (a) comparison of GnRHR mRNA expression; (b) comparison of Conexin43 mRNA expression; (c) comparison of LHCGR mRNA expression; (d) comparison of EREG mRNA expression; (e) comparison of VEGF mRNA expression. ^∗^*p* < 0.05.

**Figure 5:** The correlation between hCG and mature genes. (a) The correlation between hCG and GnRHR (*r* = 0.584). (b) The correlation between hCG and Conexin43 (*r* = 0.503). (c) The correlation between hCG and LHCGR (*r* = 0.746). (d) The correlation between hCG and EREG (*r* = 0.591). (e) The correlation between hCG and VEGF (*r* = 0.662).

**Figure 6:** Expression of PI3K/AKT/mTOR pathway-related proteins. Dot plots (a) and quantitative protein levels (b) of PI3K, AKT, and mTOR. ^∗^*p* < 0.05.

**Table 1:** Primer sequences used for RT-PCR analysis.

	Sense	Antisense
GnRHR	GGAGTTCAATCACTTGGCGT	CTTCAGCCGTGCTCTTGGTA
Conexin43	GACCACAGCTGCCTCTTCAT	CTTCAGCCGTGCTCTTGGTA
LHCGR	TGGAGAAGATGCAATGGA	GGCAATTAGCCTCTGAATGG
EREG	ACAGGCAGTCCTCAGTACAACTGTG	TGACACTTGCTCAGAGCGGA
VEGF	TGGGCCTTGCTCAGAGCGGA	GCTCACCGCCTCGGCTTGTC

**Table 2:** Comparison of general data (*n* (%)).

	Observation group (*n* = 27)	Control group (*n* = 27)	*t* or *χ*^2^	*p*
Age	28.6 ± 5.1	27.5 ± 5.4	0.770	0.445
BMI (kg/m^2^)	22.48 ± 2.51	21.96 ± 2.39	0.780	0.439
Residence			0.386	0.535
Rural	8 (29.63)	6 (22.22)		
Town	19 (70.37)	21 (77.78)		
Educational level			0.300	0.584
<High school	14 (51.85)	16 (59.26)		
≥High school	13 (48.15)	11 (40.74)		
Marital status			1.080	0.299
Married	24 (88.89)	26 (96.30)		
Unmarried	3 (11.11)	1 (3.70)		
Family medical history			2.077	0.150
Yes	2 (7.41)	0 (0.00)		
No	25 (92.59)	27 (100.00)		
Diet pill intake history			1.543	0.214
Yes	9 (33.33)	5 (18.52)		
No	18 (66.67)	22 (81.48)		
Dietary habit			0.667	0.414
Light	12 (44.44)	15 (55.56)		
Spicy	15 (55.56)	12 (44.44)		
Nationality			0.353	0.553
Han nationality	26 (96.30)	25 (92.59)		
Minority	1 (3.70)	2 (7.41)		
Smoking			1.200	0.273
Yes	6 (22.22)	3 (11.11)		
No	21 (77.78)	24 (88.89)		
Exercise habit			0.092	0.761
Yes	7 (25.93)	8 (29.63)		
No	20 (74.07)	19 (70.37)		
History of gestation			2.077	0.150
Yes	0 (0.00)	2 (7.41)		
No	27 (100.00)	25 (92.59)		
Menstruation			0.912	0.340
Normal	19 (70.37)	22 (81.48)		
Chaotic	8 (29.63)	5 (18.52)		

**Table 3:** Comparison of oocyte maturation (*n* (%)).

	Observation group	Control group	*χ* ^2^	*p*
Total MII oocytes	423	318		
Maturation rate	86.50	75.53	18.000	<0.001
Normal fertilization rate	367 (86.76)	248 (77.99)	9.902	0.002
Cleavage rate	348 (94.82)	216 (87.10)	11.620	<0.001
High-quality embryo rate	174 (47.41)	93 (37.50)	5.918	0.015

## Data Availability

The labeled dataset used to support the findings of this study are available from the corresponding author upon request.
